# Effect of incisional negative pressure therapy and conventional treatment on wound complications after orthopaedic trauma surgery: A meta‐analysis of randomized controlled studies

This article has been retracted.

**DOI:** 10.1111/iwj.14331

**Published:** 2023-08-03

**Authors:** Ping Li, Junhong Li

**Affiliations:** ^1^ Department of Orthopedics People's Hospital Affiliated of Shandong First Medical University Jinan China; ^2^ Department of Cardiac Care Unit People's Hospital Affiliated of Shandong First Medical University Jinan China

**Keywords:** deep infections, negative pressure wound therapy, superficial infections, wound dehiscence

## Abstract

The results of this meta‐analysis were applied to analyse the effects of Negative Pressure Wound Therapy (NPWT) and conventional dressings on post‐surgical outcomes after trauma in orthopaedics. Through June 2023, a full review of the literature has been carried out with the help of 4 databases, PubMed, Embase, Cochrane Library, and the Web of Science. The quality of the literature was evaluated according to the classification and exclusion criteria established for this trial, which led to an analysis of 9 related trials. The results included the injury was deeply and superficially infected, and the wound was dehiscence. The 95% confidence interval (CI) and odds ratios (OR) were computed by means of a fixed‐effect and a random‐effect model. Meta‐analyses were conducted with RevMan 5.3. There is no statistical significance between NPWT and routine therapy for deep wound infection (OR, 1.37; 95% CI, 0.82–2.27, *p* = 0.23); There was no difference in the incidence of inflammation in the wound than with conventional dressings (OR, 1.10; 95% CI, 0.84–1.45, *p* = 0.49); But NPWT was obviously superior to that of routine therapy in superficial wound infection (OR, 2.07; 95% CI, 1.32–3.25, *p* = 0.002) and wound dehiscence (OR, 2.44; 95% CI, 1.31–4.57, *p* = 0.005); But not with respect to wound exudate. therapy group, but no statistically significant difference was found with respect to wound exudation. (OR, 1.16; 95% CI, 0.86–1.57, *p* = 0.34). Given that some of the chosen trials are too small for this meta‐analysis, caution should be exercised when treating their values. More high‐quality research with a large sample is required in order to confirm the findings.

## 1 INTRODUCTION

Post‐surgical wound infections usually cause long periods of hospitalization, re‐admission and re‐surgery, which may cause patients' quality of life to deteriorate.^1^ Patients with post‐operative wound infections tend to have poorer clinical results, for example, sustained pain and delayed function recovery than others.^2^ Patients' basic health status is a risk factor for infection in orthopaedic surgery.^3^ There have been reports that Negative‐Pressure Injury Treatment (NPWT) is associated with the reduction of injury, including necrosis, infection, haematoma and hematom.^4^, ^5^ NPWT is composed of three major parts for the creation of an atmosphere of negative pressure: vacuum equipment, porous dressing and connections.^6^ NPWT decreases the amount of dead area and minimizes stress by providing a cover for the wound This improves the circulation of blood and decreases swelling, thus facilitating the healing of the wound.^7^, ^8^ It is effective in treating open wounds and healing injuries following plastic surgery. Physicians apply NPWT to patients with cardiac, abdomen and orthopaedic procedures to lower the risk of infection and speed up recovery^5^, ^8^, ^9^, ^10^, ^11^ Recent research has shown that preventive NPWT can be administered for closure of a wound following a lower extremity trauma.^12^

In an earlier meta‐analysis, which compared NPWT to standard care, there was no statistically significant difference in wound healing rates among open‐cut patients.^13^ A further meta‐analyses of NPWT versus traditional wound dressing in orthopaedic injuries showed that the incidence of deep SSI, shallow SSI, and injury dehiscences.^14^ While these findings indicate that NPWT might be a useful tool for reduction of incisional complications in orthopaedic surgical operations, there is insufficient evidence for NPWT efficacy in reduction of SSI in different types of orthopaedic operations. The purpose of this research is to confirm the results.

## 2 METHODS

### 2.1 Search strategy

From the beginning of the database until May 2023, we looked up trauma‐related surgery research in orthopaedics with PubMed, Embase, Cochrane Library, and the Web of Science. Search terms such as “orthopaedic trauma”, “negative‐pressure wound therapy”, and so on. The method of finding is illustrated in Table 1. All related data files are imported into EndNote for later processing. Furthermore, a critical review was carried out by examining the headings, summaries, and whole papers to determine the related research.

**TABLE 1:** Search strategy.

No.	Query
#1	Fracture[Title/Abstract] OR Orthopaedic trauma[Title/Abstract]
#2	Negative pressure wound therapy[Title/Abstract] OR NPWT[Title/Abstract] OR Vacuum assisted closure[Title/Abstract] OR Vacuum sealing drainage[Title/Abstract] OR VSD[Title/Abstract] OR Vacuum‐assisted closure[Title/Abstract] OR VAC[Title/Abstract] OR Sealed surface wound suction[Title/Abstract]
#3	Dressing*[Title/Abstract]
#4	Randomized OR Randomization[All Files]
#5	Incision*[All Files] OR Infection[All Files] OR Dehiscence [All Files]OR Wound complication* [All Files]OR Haemorrhage[All Files] OR Haematoma[All Files]
#6	#1 AND #2 AND #3 AND #4 AND #5

### 2.2 Information sources

Figure 1 illustrates the standard of documentation gathering for the whole study. Classification criteria are established according to participants, interventions, comparisons, outcomes and study design（PICOS） Opinion Recognition Retrieval Protocol.

**FIGURE 1:** Flow chart of the study.

The inclusion criteria were as follows:

1. Population: patients undergoing orthopaedic surgery related to trauma.
2. Intervention and Comparative Research on Post‐Operative Wound Complications Compared with conventional dressings and NPWT.
3. Design: Randomized controlled trial.

Exclusion criteria were as follows:

1. There is no comparison between NPWT and traditional dressing following orthopaedic trauma.
2. Non‐complete studies.
3. Summary, meeting, case report, review and duplication of research.

### 2.3 Data extraction

The data collected from the database were all chosen by writer Ping Li and writer Junhong Lee on the basis of the exclusion standard. The data collected in this study were the title of the main author, the date of the research, the country or province, the number of participants, and the type of research. If there is a lack of information, we will contact the authors to look for the missing information.

### 2.4 Literature quality assessment

In randomized controlled studies, we evaluated the risk of bias in accordance with the Cochrane System Review Handbook in seven areas: random‐sequence production, assignment concealment, participant and staff blindness, outcome evaluation blindness, incomplete results, selective results reporting, and other bias. For each field, the hazard ratio has been classified into three categories: Low, High, or Uncertain. “Unclear” indicates that there is not sufficient information to evaluate the risk of bias in a field. The differences were addressed by a discussion, and we were able to derive a general quality from these findings, Figure 2 and Figure 3.

**FIGURE 2:** Risk of bias diagram.

**FIGURE 3:** Risk of bias domains.

### 2.5 Reporting bias assessment

Statistical and qualitative measurements were made on the basis of Egger regression and a funnel graph that indicated the odds ratios (OR) log versus its standard error (no survey bias was taken into account if *p* ≥ 0.05).

### 2.6 Statistical analysis

The results were statistically analysed with RevMan 5.3. Estimates of the total results are given in the following forest plot. In the case of binary results, an OR was computed with 95% confidence interval (CI) (95% CI) and an intermediate result (MD) with a 95% CI. The I^2^ statistical method is employed, and the heterogeneity is thought to be high when I^2^ is above 50%. In case of substantial heterogeneity observed in meta‐analyses, random effects were employed; in other cases, fixed effects were employed. The *p* values below 0.05 were regarded as statistically significant.

## 3 RESULTS

Out of 143 related studies, nine publications were chosen to be screened for inclusion and released from 2012 to 2022. The results of those trials are presented in Table 2. Among the 3062 patients who received trauma‐type orthopaedic surgery, 1529 received negative pressure care (NPC) and 1533 received standard care.^15^, ^16^, ^17^, ^18^, ^19^, ^20^, ^21^, ^22^, ^23^ The overall sample size was between 16 and 739 individuals. Nine reviews of literature quality have been conducted, and the results are presented in Figures 2 and 3.

**TABLE 2:** Distribution characteristics of the selected studies used for meta‐analysis.

Study	Year	Country	CD	NPWT
Arti.^15^	2016	Iran	45	45
Canton.^16^	2020	Italy	49	16
Costa.^17^	2018	Britain	234	226
Costa.^18^	2020	Britain	713	739
Costa.^19^	2018	Britain	234	226
Crist.^20^	2017	Britain	33	33
Kumaar.^21^	2022	Sri Lanka	64	64
Stannard.^22^	2012	America	122	141
Wang.^23^	2019	China	39	39

NPWT levels were not significantly different from those in the routine therapy group about deep wound infection(OR, 1.37; 95% CI, 0.82–2.27, *p* = 0.23) and heterogeneity (I2 = 45%), as illustrated in Figure 4.; There was no difference between the two groups with respect to wound inflammation(OR, 1.10; 95% CI, 0.84–1.45, *p* = 0.49), as in Figure 5; But not in superficial wound infection (OR, 2.07; 95% CI, 1.32–3.25, *p* = 0.002) and wound dehiscence (OR, 2.44; 95% CI, 1.31–4.57, *p* = 0.005), NPWT is superior to routine therapy, Figure 6, Figure 7.; However, no statistically significant difference was found with respect to wound exudation (OR, 1.16; 95% CI, 0.86–1.57, *p* = 0.34) Figure 8.

**FIGURE 4:** Forest plot of the effect of deep postoperative wound infection in NPWT patients compared to controls.

**FIGURE 5:** Effect forest plot of postoperative wound inflammatory response in NPWT patients compared to control group.

**FIGURE 6:** Forest plot of the effect of superficial postoperative wound infection in NPWT patients compared to controls.

**FIGURE 7:** Forest plot of the effect of postoperative wound dehiscence in NPWT patients compared to controls.

**FIGURE 8:** Forest plot of the effect of postoperative wound ooze in NPWT patients compared to controls.

Because of certain missing data (such as sex, age, and ethnic origin), this trial could not be applied to investigate the impact of certain factors on post‐surgical trauma outcomes. There was no evidence of bias in the study by means of the quantitative Egger regression and the visualization of the funnel plot (*p* > 0.05). This is illustrated in Figures 9, 10, 11, 12 and 13. Nevertheless, the majority of nonrandomized controlled studies were considered to be of good methodology and did not have any bias in selection.

**FIGURE 9:** Funnel plot of outcomes of deep postoperative wound infection in NPWT patients compared to control group.

**FIGURE 10:** Funnel plot of outcomes of postoperative wound inflammatory response in NPWT patients compared to control group.

**FIGURE 11:** Funnel plot of outcomes of superficial postoperative wound infection in NPWT patients compared to control group.

**FIGURE 12:** Funnel plot of outcomes for post‐operative wound dehiscence in NPWT patients compared to controls.

**FIGURE 13:** Funnel plot of outcomes for post‐operative wound ooze in NPWT patients compared to control group.

## 4 DISCUSSION

Past research has demonstrated the feasibility of lowering the incidence of NPWT surgery on a biological basis.^24^ NPWT's suggested mechanism is that it allows the injury to contract, purify the extracellular fluid, and induce cellular tension, all of which is expected to speed up the healing process, thus providing an advantageous environment for angiogenesis.^25^ It also functions as a microbiological barrier, contributing to the improvement of the circulation of blood and the improvement of the oxygen supply in the body. NPWT improves the healing of the wound through the removal of excessive interstitial fluid, reduction of swelling, and promotion of growth in the open wound.^26^

Our findings are in line with earlier meta‐analyses. Past research has shown strong evidence for a significant reduction in complications associated with orthopaedic surgery with NPWT.^27^, ^28^, ^29^, ^30^, ^31^ Thus, the success of NPWT in general wound healing has prompted a number of doctors to employ NPWT in orthopaedic surgery. A meta‐analysis was performed to evaluate the occurrence of injury complications among NPWT and routine wound dressing during orthopaedic injury operations.

In this meta‐analysis, 3062 trauma orthopaedic patients were enrolled in the chosen trial, 1529 of them had SBP and 1533 received standard therapy.^15^, ^16^, ^17^, ^18^, ^19^, ^20^, ^21^, ^22^, ^23^ NPWT was associated with a reduced risk of surface injury and wound dehiscence in patients receiving trauma treatment than with conventional dressings. Strict standards should be used to treat these data throughout the course of the trial since half of the nine trials included fewer than 100 participants.

In this paper, we analysed and proved that NPWT was associated with a reduction of certain post‐surgical complications in patients undergoing an orthopaedic trauma‐type surgery, for example, a superficial wound infection or wound dehiscence. Further research is required to prove that NPWT is superior to traditional dressings in treating other post‐operative injuries. Large randomized trials are needed. Earlier research has also highlighted the problem of sample size and has come to a conclusion that is similar to this one. While it is not possible to determine if there is a strong correlation between such variations in injury complications and the results being investigated, a proper RCT trial will be necessary to investigate the impact of both post‐operative wound treatment methods on post‐surgical trauma in individuals of various ages, sexes and nationalities. Overall, NPWT has a better effect than routine dressing on the incidence of post‐operative trauma complications in trauma orthopaedics.

### 4.1 Limitations

The findings are likely to be selective because there are a number of trials that are not included in the meta‐analyses. But those that were excluded from the trial did not qualify for meta‐analyses. Furthermore, we do not have the professional knowledge to ascertain if there are other factors that affect the outcome of the study. The purpose of this research is to investigate the influence of NPWT and routine dressing on post‐operative trauma complications. Bias can be enhanced due to incomplete or inaccurate data contained in previous research. Possible sources of bias include the nutritional status of individuals as well as their race, age and gender. Furthermore, incomplete data and some unpublished work could have had an impact on the value of the studies performed.

## 5 CONCLUSION

Among those who received trauma‐type orthopaedic procedures, there was a reduced risk of surface wound infection and injury dehiscence after the operation than with traditional dressings. Care should, however, be taken with regard to their values, since there are few identified trials for meta‐analyses.

## CONFLICT OF INTEREST STATEMENT

The authors declare that there is no conflict of interest.

## Data Availability

Data available on request from the authors.

## References

[1] Alverdy JC , Hyman N , Gilbert J . Re‐examining causes of surgical site infections following elective surgery in the era of asepsis. Lancet Infect Dis. 2020;20(3):e38‐e43.10.1016/S1473-3099(19)30756-XPMC801915432006469

[2] Zhou J , Wang R , Huo X , Xiong W , Kang L , Xue Y . Incidence of surgical site infection after spine surgery: a systematic review and meta‐analysis. Spine (Phila Pa 1976). 2020;45(3):208‐216.3146497210.1097/BRS.0000000000003218

[3] Shao J , Zhang H , Yin B , Li J , Zhu Y , Zhang Y . Risk factors for surgical site infection following operative treatment of ankle fractures: a systematic review and meta‐analysis. Int J Surg. 2018;56:124‐132.2992902210.1016/j.ijsu.2018.06.018

[4] Huang C , Leavitt T , Bayer LR , Orgill DP . Effect of negative pressure wound therapy on wound healing. Curr Probl Surg. 2014;51(7):301‐331.2493507910.1067/j.cpsurg.2014.04.001

[5] Colli A , Camara ML . First experience with a new negative pressure incision management system on surgical incisions after cardiac surgery in high risk patients. J Cardiothorac Surg. 2011;6:160.2214564110.1186/1749-8090-6-160PMC3305521

[6] Whitehouse JD , Friedman ND , Kirkland KB , Richardson WJ , Sexton DJ . The impact of surgical‐site infections following orthopedic surgery at a community hospital and a university hospital: adverse quality of life, excess length of stay, and extra cost. Infect Control Hosp Epidemiol. 2002;23(4):183‐189.1200223210.1086/502033

[7] Stannard JP , Singanamala N , Volgas DA . Fix and flap in the era of vacuum suction devices: what do we know in terms of evidence based medicine? Injury. 2010;41(8):780‐786.2047101210.1016/j.injury.2009.08.011

[8] Suzuki T , Minehara A , Matsuura T , Kawamura T , Soma K . Negative‐pressure wound therapy over surgically closed wounds in open fractures. J Orthop Surg (Hong Kong). 2014;22(1):30‐34.2478160910.1177/230949901402200109

[9] Stannard JP , Gabriel A , Lehner B . Use of negative pressure wound therapy over clean, closed surgical incisions. Int Wound J. 2012;9(Suppl 1):32‐39.2272713810.1111/j.1742-481X.2012.01017.xPMC7950357

[10] Hudson DA , Adams KG , Van Huyssteen A , Martin R , Huddleston EM . Simplified negative pressure wound therapy: clinical evaluation of an ultraportable, no‐canister system. Int Wound J. 2015;12(2):195‐201.2364773710.1111/iwj.12080PMC7950749

[11] Yang CC , Chang DS , Webb LX . Vacuum‐assisted closure for fasciotomy wounds following compartment syndrome of the leg. J Surg Orthop Adv. 2006;15(1):19‐23.16603108

[12] Cooper HJ , Bas MA . Closed‐incision negative‐pressure therapy versus antimicrobial dressings after revision hip and knee surgery: a comparative study. J Arthroplast. 2016;31(5):1047‐1052.10.1016/j.arth.2015.11.01026712346

[13] Iheozor‐Ejiofor Z , Newton K , Dumville JC , Costa ML , Norman G , Bruce J . Negative pressure wound therapy for open traumatic wounds. Cochrane Database Syst Rev. 2018;7(7):CD012522.2996952110.1002/14651858.CD012522.pub2PMC6513538

[14] Wang C , Zhang Y , Qu H . Negative pressure wound therapy for closed incisions in orthopedic trauma surgery: a meta‐analysis. J Orthop Surg Res. 2019;14(1):427.3182921710.1186/s13018-019-1488-zPMC6907184

[15] Arti H , Khorami M , Ebrahimi‐Nejad V . Comparison of negative pressure wound therapy (NPWT) &conventional wound dressings in the open fracture wounds. Pak J Med Sci. 2016;32(1):65‐69.2702234710.12669/pjms.321.8568PMC4795891

[16] Canton G , Fattori R , Pinzani E , Monticelli L , Ratti C , Murena L . Prevention of postoperative surgical wound complications in ankle and distal tibia fractures: results of incisional negative pressure wound therapy. Acta Biomed. 2020;91(14‐S):e2020006.10.23750/abm.v91i14-S.10784PMC794468333559636

[17] Costa ML , Achten J , Bruce J , et al. Negative‐pressure wound therapy versus standard dressings for adults with an open lower limb fracture: the WOLLF RCT. Health Technol Assess (Winch Eng). 2018;22(73):1‐162.10.3310/hta22730PMC632206130573002

[18] Costa ML , Achten J , Bruce J , et al. Effect of negative pressure wound therapy vs standard wound management on 12‐month disability among adults with severe open fracture of the lower limb the wollf randomized clinical trial. JAMA ‐ J Am Med Assoc. 2018;319(22):2280‐2288.10.1001/jama.2018.6452PMC658350429896626

[19] Costa ML , Achten J , Knight R , et al. Negative‐pressure wound therapy compared with standard dressings following surgical treatment of major trauma to the lower limb: the WHiST RCT. Health Technol Assess (Winch Eng). 2020;24(38):1‐86.10.3310/hta24380PMC745706132821038

[20] Crist BD , Oladeji LO , Khazzam M , Della Rocca GJ , Murtha YM , Stannard JP . Role of acute negative pressure wound therapy over primarily closed surgical incisions in acetabular fracture ORIF: a prospective randomized trial. Injury. 2017;48(7):1518‐1521.2847799210.1016/j.injury.2017.04.055

[21] Kumaar A , Shanthappa AH , Ethiraj P . A comparative study on efficacy of negative pressure wound therapy versus standard wound therapy for patients with compound fractures in a tertiary care hospital. Cureus. 2022;14(4):e23727.3550976710.7759/cureus.23727PMC9060726

[22] Stannard JP , Volgas DA , McGwin G 3rd , et al. Incisional negative pressure wound therapy after high‐risk lower extremity fractures. J Orthop Trauma. 2012;26(1):37‐42.2180441410.1097/BOT.0b013e318216b1e5

[23] Wang Z . The effects of vacuum sealing drainage on improving the efficacy of reducing wound infection and lower extremity deep venous thrombosis in patients with orthopedic trauma. Int J Clin Exp Med. 2019;12(12):13839‐13846.

[24] Nolff MC , Meyer‐Lindenberg A . Negative pressure wound therapy (NPWT) in small animal medicine. Mechanisms of action, applications and indications. Tierarztl Prax Ausg K Kleintiere Heimtiere. 2016;44(1):26‐37. quiz 8.2683072510.15654/TPK-150957

[25] Namgoong S , Han SK . Status of wound management in Korea. Wound Repair Regen. 2018;26(Suppl 1):S3‐S8.2885739910.1111/wrr.12576

[26] Normandin S , Safran T , Winocour S , et al. Negative pressure wound therapy: mechanism of action and clinical applications. Semin Plast Surg. 2021;35(3):164‐170.3452686410.1055/s-0041-1731792PMC8432996

[27] Liu X , Zhang H , Cen S , Huang F . Negative pressure wound therapy versus conventional wound dressings in treatment of open fractures: a systematic review and meta‐analysis. Int J Surg. 2018;53:72‐79.2955553010.1016/j.ijsu.2018.02.064

[28] Gao J , Wang Y , Song J , Li Z , Ren J , Wang P . Negative pressure wound therapy for surgical site infections: a systematic review and meta‐analysis. J Adv Nurs. 2021;77(10):3980‐3990.3390555210.1111/jan.14876

[29] Grant‐Freemantle MC , Ryan EJ , Flynn SO , et al. The effectiveness of negative pressure wound therapy versus conventional dressing in the treatment of open fractures: a systematic review and meta‐analysis. J Orthop Trauma. 2020;34(5):223‐230.3207989010.1097/BOT.0000000000001750

[30] Norman G , Goh EL , Dumville JC , et al. Negative pressure wound therapy for surgical wounds healing by primary closure. Cochrane Database Syst Rev. 2020;6:CD009261.3254264710.1002/14651858.CD009261.pub6PMC7389520

[31] Kuo FC , Hsu CW , Tan TL , Lin PY , Tu YK , Chen PC . Effectiveness of different wound dressings in the reduction of blisters and periprosthetic joint infection after Total joint arthroplasty: a systematic review and network meta‐analysis. J Arthroplast. 2021;36(7):2612‐2629.10.1016/j.arth.2021.02.04733707123

